# The Top 50 Articles on Knee Posterolateral Corner Injuries

**DOI:** 10.1016/j.asmr.2022.06.017

**Published:** 2022-08-20

**Authors:** Andre Perez-Chaumont, Tolulope Ramos, Wendell W. Cole, Michaela A. Stamm, Mary K. Mulcahey

**Affiliations:** a Department of Orthopaedic Surgery New Orleans, Louisiana, U.S.A.; b Tulane University School of Medicine New Orleans, Louisiana, U.S.A.

## Abstract

**Purpose:**

To identify and characterize the most cited publications in orthopaedic research related to posterolateral corner (PLC) injuries of the knee.

**Methods:**

The Science Citation Index Expanded was queried for PLC injury articles. The 50 most-cited studies from 1976 to 2021 were selected. Article characteristics, including number of citations, citation density, year of publication, source journal, country of origin, article type, article subtype, and level of evidence, were analyzed.

**Results:**

The number of citations for individual articles ranged from 47 to 205. The 50 most cited articles were published in 16 journals. Eleven of the 50 articles (22%) were published in *Arthroscopy—The Journal of Arthroscopic and Related Surgery*. The largest proportion of the articles (n = 22, 44%) were classified as clinical, with the rest classified as reviews (n = 15, 30%), and basic science research (n = 13, 26%). The most common level of evidence for clinical articles was IV (14/22, 63.6%). Nine countries contributed to the top 50 articles, with the majority published in the United States (n = 35, 70%).

**Conclusions:**

In the last 20 years, papers published on the diagnosis and surgical management of PLC injuries have a high citation frequency. Future high-quality research is needed to establish best-practice guidelines for the management of PLC injuries due to the low overall level of evidence of existing clinical studies.

**Clinical Relevance:**

This research provides a comprehensive list for practitioners and may help educators identify articles to include in the curriculum for residents and fellows.

The posterolateral corner (PLC) of the knee was once referred to as the “dark side” of the knee due to the historically limited understanding of PLC anatomy and the poor outcomes associated with injuries to this area.^1^ The PLC is a complex anatomical area that includes the lateral collateral ligament, popliteus tendon, and the popliteofibular ligament.^2^ Injuries to the PLC often go undiagnosed and were previously considered to be a rare condition; however, they recently have been reported to be present in up to 16% of knee injuries.^3^ PLC injuries most often occur in conjunction with injury to other structures of the knee. Injury to the PLC of the knee is particularly associated with posterior cruciate ligament (PCL) injury, followed by anterior cruciate ligament (ACL) injury. Up to 70% of PCL tears show concomitant damage to the PLC. While the identification of PLC injuries is sometimes difficult, diagnosis is crucial to optimizing surgical and clinical outcomes in these patients.^4^ If left untreated, these injuries can lead to chronic pain and instability, early development of osteoarthritis, and failure of cruciate ligament reconstructions.^2^^,^^3^^,^^5^

Citation impact, or how many times a scientific publication is cited in the literature, can be used as an indicator of an article’s influence in a particular field of study.^6^^,^^7^ Although the number of times an article has been cited is not the only factor determining the importance an article has on its area of medical expertise, it can be useful for indicating the landmark scientific investigations or “citation classics” in a particular field.^8^ Analyses of most-cited papers can prove valuable to medical educators by helping identify articles of particular importance that may warrant inclusion in their trainees’ reading curriculum.

In 2011, Lefaivre et al.^9^ published a citation analysis of the seminal works in orthopaedic surgery, and multiple similar studies have since investigated the most influential papers related to various orthopaedic subspecialties and conditions.^7^^,^^9^, ^10^, ^11^, ^12^, ^13^ The purpose of this study was to identify and characterize the most-cited publications in orthopaedic research related to PLC injuries of the knee. It was hypothesized that there would be many highly-cited articles related to PLC injuries published in the last 2 decades and that the minority would present high levels of evidence.

## Methods

In accordance with previously described methods in similar studies,^7^^,^^9^, ^10^, ^11^, ^12^, ^13^, ^14^ a systematic search of the Science Citation Index Expanded database (v5.35; Thomson Reuters) was performed by one author (A.P.) in August 2021 to identify articles related to PLC injuries. Using the Advanced Search tool, “All Databases” was selected and the parameters of the search was set to include journals published from 1976 to 2021 listed under the Web of Science categories "Orthopedics" and “Sports Science.” The following search terms were used: “posterolateral corner,” “posterolateral corner injuries,” “PLC injury,” and “PLC repair.” The results were sorted according to the total number of citations. In cases in which 2 or more articles had the same total number of citations, ranking order was determined using citation density. After screening the abstracts of each result to ensure that the material was related to PLC injuries of the knee, the 50 most-cited articles were selected for analysis.

For each of the articles, the following characteristics were recorded: total number of citations, citation density, year of publication, source journal, and country of origin. All data were extracted, synthesized, and recorded using Microsoft Excel (version 16.0, Redmond, WA). Citation density was defined as the number of citations per year since the date of publication. Country of origin was determined by the corresponding author’s country of origin. The articles were then characterized by scientific type including clinical, basic science, or review/expert opinion. Anatomic, cadaveric, and biomechanical studies performed in a laboratory setting were included in the “Basic Science” category, whereas nonsystematic reviews and surgical technique articles were included in the “Review/Expert Opinion” category. Clinical articles were further subtyped as either therapeutic, prognostic, or diagnostic. The *Journal of Bone and Joint Surgery* (*JBJS*) guidelines were used to evaluate the level of evidence for each clinical article.^15^

## Results

The 50 most-cited publications relating to PLC injuries of the knee were cited a total of 4,235 times by 1,752 articles in the literature. A list of the 10 most-cited articles, their respective total number of citations, and citation densities can be found in Table 1.^14^^,^^16^, ^17^, ^18^, ^19^, ^20^, ^21^, ^22^, ^23^, ^24^ A complete list of the 50 most-cited articles can be found in Appendix Table 1, available at www.arthroscopyjournal.org. The number of citations for individual articles ranged from 47 to 205 (mean 84.7; standard deviation ± 40.2) and citation densities ranged from 2.16 to 15.77 (mean 5.56; standard deviation ± 2.9). The article “Decision Making in the Multiligament-Injured Knee: An Evidence-Based Systematic Review” by Levy et al.^16^ had the highest citation total (205) and highest citation density (15.77) of the publications included in this study.

**Table 1:** The Top 10 Cited Articles on Posterolateral Corner Injuries of the Knee.

Rank	Article	Number of Citations	Citation Density
1	Levy BA, Dajani KA, Whelan DB, et al. Decision making in the multiligament-injured knee: An evidence-based systematic review. *Arthroscopy* 2009;25:430-438.^16^	205	15.77
2	Stannard JP, Brown SL, Farris RC, et al. The posterolateral corner of the knee: Repair versus reconstruction. *Am J Sports Med* 2005;33:881-888^14^	196	11.53
3	Covey DC. Injuries of the posterolateral corner of the knee. *J Bone Joint Surg Am* 2001;83:106-118^17^	176	8.38
4	Levy BA, Dajani KA, Morgan JA, et al. Repair versus reconstruction of the fibular collateral ligament and posterolateral corner in the multiligament-injured knee. *Am J Sports Med* 2010;38:804-809^18^	154	12.83
5	Gardner MJ, Yacoubian S, Geller D, et al. The incidence of soft tissue injury in operative tibial plateau fractures: A magnetic resonance imaging analysis of 103 patients. *J Orthop Trauma* 2005;19:79-84^19^	145	8.53
6	Fanelli GC, Orcutt DR, Edson CJ. The multiple-ligament injured knee: Evaluation, treatment, and results. *Arthroscopy* 2005;21:471-486^20^	138	8.12
7	Fanelli GC, Edson CJ. Combined posterior cruciate ligament-posterolateral reconstructions with Achilles tendon allograft and biceps femoris tendon tenodesis: 2- to 10-year follow-up. *Arthroscopy* 2004;20:339-345^21^	128	7.11
8	LaPrade RF, Heikes C, Bakker AJ, et al. The reproducibility and repeatability of varus stress radiographs in the assessment of isolated fibular collateral ligament and grade-III posterolateral knee injuries. An in vitro biomechanical study. *J Bone Joint Surg Am* 2008;90:2069-2076^22^	125	8.93
9	Levy BA, Fanelli GC, Whelan DB, et al. Controversies in the treatment of knee dislocations and multiligament reconstruction. *J Am Acad Orthop Surg* 2009;17:197-206^23^	123	9.46
10	LaPrade RF, Wentorf FA, Fritts H, et al. A prospective magnetic resonance imaging study of the incidence of posterolateral and multiple ligament injuries in acute knee injuries presenting with a hemarthrosis. *Arthroscopy* 2007;23:1341-1347^24^	112	7.47

The top 50 articles were published in 16 different journals (Table 2). The journals that published the largest number of articles were *Arthroscopy—The Journal of Arthroscopic and Related Surgery* (n = 11, 22%), followed by *The American Journal of Sports Medicine* (*AJSM*) (n = 10, 20%), and *JBJS* (n = 6, 12%). The publication years ranged from 1994 to 2016 (Fig 1). 2005, 2006, and 2008 were the years in which the highest number of articles were published with 9, 6, and 6 publications respectively. Nine countries of origin were identified for the 50 most-cited articles (Table 3). The majority were published in the United States (n = 35, 70%), followed by Greece (n = 3, 6%), Germany (n = 2, 4%), and South Korea (n = 2, 4%).

**Table 2:** A Breakdown of Journals in Which the Top 50 Articles Related to PLC Injuries Were Published

Journal	No. of Articles	% of Articles
*Arthroscopy - The Journal of Arthroscopic and Related Surgery*	11	22%
*American Journal of Sports Medicine*	10	20%
*Journal of Bone and Joint Surgery - American Volume*	6	12%
*American Journal of Roentgenology*	3	6%
*Journal of Bone and Joint Surgery - British Volume*	3	6%
*Knee Surgery, Sports Traumatology, Arthroscopy*	3	6%
*Sports Medicine and Arthroscopy Review*	3	6%
*Clinics in Sports Medicine*	2	4%
*Journal of the American Academy of Orthopaedic Surgeons*	2	4%
*Archives of Bone and Joint Surgery*	1	2%
*Archives of Orthopaedic and Trauma Surgery*	1	2%
*Instructional Course Lectures*	1	2%
*Journal of Orthopaedic & Sports Physical Therapy*	1	2%
*Journal of Orthopaedic Trauma*	1	2%
*Radiographics*	1	2%
*Skeletal Radiology*	1	2%

PLC, posterolateral corner.

**Fig 1:** Breakdown of top 50 articles by year published.

**Table 3:** Countries of Origin for the 50 Most-Cited Articles on PLC Injuries

Country of Origin	No. of Articles	% of Articles
United States	35	70%
Greece	3	6%
Germany	2	4%
South Korea	2	4%
Australia	1	2%
Taiwan	1	2%
Austria	1	2%
Canada	1	2%
Netherlands	1	2%

PLC, posterolateral corner.

Of the top 50 publications on PLC injury, 22 (44%) were classified as “Clinical,” 15 (30%) as “Review/Expert Opinion,” and 13 (26%) as “Basic Science.” The majority of the clinical articles were subclassified as “Clinical–Therapeutic” (15/22, 68.2%). Most clinical articles (14/22, 63.6%) met the standard for Level IV evidence. No studies presented Level I evidence; 22.7% (5/22), 9% (2/22), and 4.5% (1/22) of articles fit criteria for Levels II, III, and V evidence, respectively (Fig 2).

**Fig 2:** Number of clinical articles by Level of Evidence.

## Discussion

This study identified the 50 most-cited articles on PLC injuries, which were cited a combined total of 4,235 times. Levy et al. 2009^16^ was the most-cited article (205 citations) with the highest citation density (15.77 citations per year), and the top 10 articles were each cited at least 112 times. Most of the included publications presented Level IV evidence. Very few publications were Level II and III studies, and none were Level I. The journals that published the largest number of most-cited articles were *Arthroscopy* (n = 11, 22%), followed by *AJSM* (n = 10, 20%), and *JBJS* (n = 6, 12%). Of the 9 countries contributing to the top 50 articles, 35 (70%) were in the United States, 7 (14%) were in Europe, and the remaining 8 (16%) originated outside the United States and Europe.

Levy et al. 2009^16^ was cited 205 times with 15.77 citations per year, making it the article with the highest citation total and density. The top 10 articles were each cited at least 112 times. These numbers are lower compared with citations for articles on other orthopaedic topics such as ACL reconstruction or total-joint arthroplasty.^12^^,^^25^ Vielgut et al.^12^ reported on the 50 most-cited papers in ACL injury and noted that the top article was cited 1,624 times, with the top 10 articles each being cited at least 601 times. Similarly, Holzer and Holzer^25^ found that the top article on hip and knee arthroplasty was cited 2,495 times and the top 10 articles were each cited at least 580 times. Research involving PLC injuries may have lower citation numbers due to other sports injuries such as ACL tears being far more common, the more recent recognition of the importance of properly diagnosing and treating these injuries, and insufficient knowledge of the related anatomy and biomechanics.

Among the most-cited clinical articles related to PLC injuries, very few were Level II (23%) and Level III (9%) evidence, whereas the majority (63.6%) were Level IV evidence. There were no articles of Level I evidence. Twenty-two of the 50 articles (44%) were classified as clinical, with 14 of the 22 (63.6%) classified as Level IV studies. Similarly, Holzer and Holzer^25^ evaluated the most-cited articles in hip and knee arthroplasty and found that 72% of (23/32) of clinical papers were Level IV evidence.^17^ In their citation analysis of articles related to ACL injury, Vielgut et al.^12^ reported a majority of Level II (10/14, 71.4%) and III (3/14, 21.4%) evidence in the clinical science and outcome categories.

Twenty-two (44%) of the top 50 cited articles related to PLC injuries were classified as clinical, with 15 of the 22 articles (68.2%) subclassified as “clinical–therapeutic,” similar to the results of other studies.^11^^,^^13^ This suggests that surgeons are interested in understanding the complications, benefits, and outcomes of different surgical techniques used for the treatment of PLC injuries. Although there are several techniques for the surgical management of PLC injuries, the LaPrade technique of anatomic reconstruction using an Achilles tendon allograft is now considered the gold standard.^26^ In addition, since PLC injuries often occur in combination with injury to the PCL or ACL, PLC and cruciate ligament reconstruction may be performed in combination.^27^ As awareness of PLC injuries and related sequelae has increased, so has research into which treatment modality is most effective. The results of this study demonstrate that the most influential clinical articles related to PLC injury are studies that inform treatment and rehabilitation. However, existing clinical studies present overall low levels of evidence and inconsistencies in surgical treatment. Future high-quality investigations are needed for sound evidence-based recommendations to be made regarding the management of PLC injuries.

The journals that published the largest number of most-cited articles were *Arthroscopy* (n = 11, 22%), followed by *AJSM* (n = 10, 20%), and *JBJS* (n= 6, 12%). The same journals have been similarly identified in recent citation analyses. In their study involving the most cited articles in shoulder arthroscopic surgery, Moore et al.^28^ also found *Arthroscopy* to be the publisher of the largest number of included studies, whereas *AJSM* published the highest number of most cited articles related to ACL injury.

Of the 9 countries contributing to the top 50 articles, 35 (70%) were from the United States, 7 (14%) were from Europe, and the remaining 8 (16%) originated outside the United States and Europe. These results are similar to trends identified in other citation analyses involving orthopaedic literature. Studies discussing the most cited articles related to ACL injuries, knee research, hip and knee arthroplasty, and shoulder arthroplasty also reported that the largest percentage of the articles in their respective studies originated from within the United States.^10^^,^^12^^,^^25^^,^^28^

Although this study may not include every publication that has influenced understanding of PLC injures, this citation analysis allowed the identification and characterization of the commonly referenced research published on the topic. This list may be beneficial for practitioners to reference and help educators identify articles to include in the curriculum for residents and fellows.

### Limitations

This study is not without limitations. One important limitation is that the articles were primarily ranked on the basis of cumulative citations; thus, newer articles with high annual citation rates may have been missed. Furthermore, our search was limited to the Web of Science database. Articles from sources including digital media, textbooks, and oral lectures as well as those published in non-index journals are not included in the database. Although citation impact frequently has been used as a marker of an article’s academic influence, this list should not be considered wholly comprehensive, given that the Web of Science only investigates citation number and density as measures of impact.^6^^,^^7^ The number of citations for a specific article can also be easily influenced by many factors including self-citations, date of publication, popularity of subject, journal prestige, and the number of authors.^20^ Although the articles included in this study may be the most cited, our study does not report the quality of the articles mentioned. Lastly, this study provides only a summary of the top 50 cited articles related to PLC injuries on the day of the search. Additional impactful articles on PLC injuries may have been published since this search was conducted; however, this is mitigated by the fact that most of the included publications were published before 2012.

## Conclusions

In the last 20 years, papers published on the diagnosis and surgical management of PLC injuries have a high citation frequency. However, the overall level of evidence of existing clinical studies pertaining to PLC injuries is low. Future high-quality clinical research is needed to address inconsistencies in surgical treatment and establish best-practice guidelines for the management of these injuries.

## Figures and Tables

**Appendix Table 1:** The Top 50 Cited Articles on Posterolateral Corner Injuries of the Knee

Rank	Article	Number of Citations	Citation Density
1	Levy BA, Dajani KA, Whelan DB, et al. Decision making in the multiligament-injured knee: An evidence-based systematic review. *Arthroscopy* 2009;25:430-438.	205	15.77
2	Stannard JP, Brown SL, Farris RC, et al. The posterolateral corner of the knee: Repair versus reconstruction. *Am J Sports Med* 2005;33:881-888.	196	11.53
3	Covey DC. Injuries of the posterolateral corner of the knee. *J Bone Joint Surg Am* 2001;83:106-118.	176	8.38
4	Levy BA, Dajani KA, Morgan JA, et al. Repair versus reconstruction of the fibular collateral ligament and posterolateral corner in the multiligament-injured knee. *Am J Sports Med* 2010;38:804-809.	154	12.83
5	Gardner MJ, Yacoubian S, Geller D, et al. The incidence of soft tissue injury in operative tibial plateau fractures: A magnetic resonance imaging analysis of 103 patients. *J Orthop Trauma*. 2005;19:79-84.	145	8.53
6	Fanelli GC, Orcutt DR, Edson CJ. The multiple-ligament injured knee: Evaluation, treatment, and results. *Arthroscopy* 2005;21:471-486.	138	8.12
7	Fanelli GC, Edson CJ. Combined posterior cruciate ligament-posterolateral reconstructions with Achilles tendon allograft and biceps femoris tendon tenodesis: 2- to 10-year follow-up. *Arthroscopy* 2004;20:339-345.	128	7.11
8	LaPrade RF, Heikes C, Bakker AJ, et al. The reproducibility and repeatability of varus stress radiographs in the assessment of isolated fibular collateral ligament and grade-III posterolateral knee injuries. An in vitro biomechanical study. *J Bone Joint Surg Am* 2008;90:2069-2076.	125	8.93
9	Levy BA, Fanelli GC, Whelan DB, et al. Controversies in the treatment of knee dislocations and multiligament reconstruction. *J Am Acad Orthop Surg* 2009;17:197-206.	123	9.46
10	LaPrade RF, Wentorf FA, Fritts H, et al. A prospective magnetic resonance imaging study of the incidence of posterolateral and multiple ligament injuries in acute knee injuries presenting with a hemarthrosis. *Arthroscopy* 2007;23:1341-1347.	112	7.47
11	Veltri DM, Warren RF. Operative treatment of posterolateral instability of the knee. *Clin Sports Med* 1994;13:615-627.	110	3.93
12	LaPrade RF, Johansen S, Agel J, et al. Outcomes of an anatomic posterolateral knee reconstruction. *J Bone Joint Surg Am* 2010;92:16-22.	106	8.83
13	Shahane SA, Ibbotson C, Strachan R, et al. The popliteofibular ligament. An anatomical study of the posterolateral corner of the knee. *J Bone Joint Surg Br* 1999;81:636-642.	105	4.57
14	Tzurbakis M, Diamantopoulos A, Xenakis T, et al. Surgical treatment of multiple knee ligament injuries in 44 patients: 2-8 years follow-up results. *Knee Surg Sports Traumatol Arthrosc* 2006;14:739-749.	104	6.5
15	Veltri DM, Warren RF. Anatomy, biomechanics, and physical findings in posterolateral knee instability. *Clin Sports Med* 1994;13:599-614.	104	3.71
16	Geeslin AG, LaPrade RF. Outcomes of treatment of acute grade-III isolated and combined posterolateral knee injuries: A prospective case series and surgical technique. *J Bone Joint Surg Am* 2011;93:1672-1683.	101	9.18
17	Fanelli GC, Larson RV. Practical management of posterolateral instability of the knee. *Arthroscopy* 2002;18:1-8.	96	4.8
18	Sekiya JK, Whiddon DR, Zehms CT, et al. A clinically relevant assessment of posterior cruciate ligament and posterolateral corner injuries. Evaluation of isolated and combined deficiency. *J Bone Joint Surg Am* 2008;90:1621-1627.	91	6.5
19	Stannard JP, Brown SL, Robinson JT, et al. Reconstruction of the posterolateral corner of the knee. *Arthroscopy* 2005;21:1051-1059.	90	5.29
20	Hayes CW, Brigido MK, Jamadar DA, et al. Mechanism-based pattern approach to classification of complex injuries of the knee depicted at MR imaging. *Radiographics* 2000;20 Spec No:S121-34.	89	4.05
21	Arthur A, LaPrade RF, Agel J. Proximal tibial opening wedge osteotomy as the initial treatment for chronic posterolateral corner deficiency in the varus knee: A prospective clinical study. *Am J Sports Med* 2007;35:1844-1850.	86	5.73
22	Strobel MJ, Schulz MS, Petersen WJ, et al. Combined anterior cruciate ligament, posterior cruciate ligament, and posterolateral corner reconstruction with autogenous hamstring grafts in chronic instabilities. *Arthroscopy* 2006;22:182-192.	76	4.75
23	Huang GS, Yu JS, Munshi M, et al. Avulsion fracture of the head of the fibula (the "arcuate" sign): MR imaging findings predictive of injuries to the posterolateral ligaments and posterior cruciate ligament. *AJR Am J Roentgenol* 2003;180:381-387.	75	3.95
24	Ranawat A, Baker CL, III, Henry S, et al. Posterolateral corner injury of the knee: Evaluation and management. *J Am Acad Orthop Surg* 2008;16:506-518.	67	4.79
25	Albright JP, Brown AW. Management of chronic posterolateral rotatory instability of the knee: Surgical technique for the posterolateral corner sling procedure. *Instr Course Lect* 1998;47:369-378.	67	2.79
26	McCarthy M, Camarda L, Wijdicks CA, et al. Anatomic posterolateral knee reconstructions require a popliteofibular ligament reconstruction through a tibial tunnel. *Am J Sports Med* 2010;38:1674-1681.	65	5.42
27	Nau T, Chevalier Y, Hagemeister N, et al. Comparison of 2 surgical techniques of posterolateral corner reconstruction of the knee. *Am J Sports Med* 2005;33:1838-1845.	65	3.82
28	Munshi M, Pretterklieber ML, Kwak S, et al. MR imaging, MR arthrography, and specimen correlation of the posterolateral corner of the knee: An anatomic study. *AJR Am J Roentgenol* Apr 2003;180:1095-1101.	65	3.42
29	Zantop T, Schumacher T, Diermann N, et al. Anterolateral rotational knee instability: Role of posterolateral structures. *Arch Orthop Trauma Surg* 2007;127:743-752.	63	4.2
30	Yoon KH, Bae DK, Ha JH, et al. Anatomic reconstructive surgery for posterolateral instability of the knee. *Arthroscopy* Feb 2006;22:159-165.	62	3.88
31	Lee J, Papakonstantinou O, Brookenthal KR, et al. Arcuate sign of posterolateral knee injuries: Anatomic, radiographic, and MR imaging data related to patterns of injury. *Skeletal Radiol* 2003;32:619-627.	61	3.21
32	Fanelli GC, Stannard JP, Stuart MJ, et al. Management of complex knee ligament injuries. *J Bone Joint Surg Am* 2010;92:2235-2246.	60	5
33	Sanchez AR, 2nd, Sugalski MT, LaPrade RF. Anatomy and biomechanics of the lateral side of the knee. *Sports Med Arthrosc Rev* 2006;14:2-11.	57	3.56
34	Azar FM, Brandt JC, Miller RH, III, et al. Ultra-low-velocity knee dislocations. *Am J Sports Med* 2011;39:2170-2174.	56	5.09
35	Brinkman JM, Schwering PJ, Blankevoort L, et al. The insertion geometry of the posterolateral corner of the knee. *J Bone Joint Surg Br* 2005;87:1364-1368.	56	3.29
36	LaPrade RF, Hamilton CD, Engebretsen L. Treatment of acute and chronic combined anterior cruciate ligament and posterolateral knee ligament injuries. *Sports Med Arthrosc Rev* 1997;5:91-99.	54	2.16
37	Diamantopoulos A, Tokis A, Tzurbakis M, et al. The posterolateral corner of the knee: Evaluation under microsurgical dissection. *Arthroscopy* 2005;21:826-833.	53	3.12
38	Geeslin AG, Moulton SG, LaPrade RF. A systematic review of the outcomes of posterolateral corner knee injuries, part 1: Surgical treatment of acute injuries. *Am J Sports Med* 2016;44:1336-1342.	52	8.67
39	Wilson WT, Deakin AH, Payne AP, et al. Comparative analysis of the structural properties of the collateral ligaments of the human knee. *J Orthop Sports Phys Ther* 2012;42:345-351.	52	5.2
40	Vinson EN, Major NM, Helms CA. The posterolateral corner of the knee. *AJR Am J Roentgenol* 2008;190:449-458.	52	3.71
41	Cooper JM, McAndrews PT, LaPrade RF. Posterolateral corner injuries of the knee: Anatomy, diagnosis, and treatment. *Sports Med Arthrosc Rev* 2006;14:213-220.	52	3.25
42	Sekiya JK, Haemmerle MJ, Stabile KJ, et al. Biomechanical analysis of a combined double-bundle posterior cruciate ligament and posterolateral corner reconstruction. *Am J Sports Med* 2005;33:360-369.	52	3.06
43	Apsingi S, Nguyen T, Bull AM, et al. Control of laxity in knees with combined posterior cruciate ligament and posterolateral corner deficiency: Comparison of single-bundle versus double-bundle posterior cruciate ligament reconstruction combined with modified Larson posterolateral corner reconstruction. *Am J Sports Med* 2008;36:487-494.	51	3.64
44	Nyland J, Hester P, Caborn DN. Double-bundle posterior cruciate ligament reconstruction with allograft tissue: 2-year postoperative outcomes. *Knee Surg Sports Traumatol Arthrosc* 2002;10:274-279.	51	2.55
45	Markolf KL, Graves BR, Sigward SM, et al. How well do anatomical reconstructions of the posterolateral corner restore varus stability to the posterior cruciate ligament-reconstructed knee? *Am J Sports Med* 2007;35:1117-1122.	49	3.27
46	Chahla J, Moatshe G, Dean CS, et al. Posterolateral corner of the knee: Current concepts. *Arch Bone Joint Surg* 2016;4:97-103.	48	8
47	Jung YB, Jung HJ, Kim SJ, et al. Posterolateral corner reconstruction for posterolateral rotatory instability combined with posterior cruciate ligament injuries: Comparison between fibular tunnel and tibial tunnel techniques. *Knee Surg Sports Traumatol Arthrosc* 2008;16:239-248.	48	3.43
48	Khanduja V, Somayaji HS, Harnett P, et al. Combined reconstruction of chronic posterior cruciate ligament and posterolateral corner deficiency. A two- to nine-year follow-up study. *J Bone Joint Surg Br* 2006;88:1169-1172.	48	3
49	Schechinger SJ, Levy BA, Dajani KA, et al. Achilles tendon allograft reconstruction of the fibular collateral ligament and posterolateral corner. *Arthroscopy* 2009;25:232-242.	47	3.62
50	Arciero RA. Anatomic posterolateral corner knee reconstruction. *Arthroscopy* 2005;21:1147.	47	2.76

MR, magnetic resonance.

## Supplementary Data

ICMJE author disclosure forms
